# Epstein-Barr Virus Nuclear Antigen 3C Stabilizes Gemin3 to Block p53-mediated Apoptosis

**DOI:** 10.1371/journal.ppat.1002418

**Published:** 2011-12-08

**Authors:** Qiliang Cai, Yi Guo, Bingyi Xiao, Shuvomoy Banerjee, Abhik Saha, Jie Lu, Tina Glisovic, Erle S. Robertson

**Affiliations:** 1 Department of Microbiology and the Tumor Virology Program, Abramson Comprehensive Cancer Center, Perelman School of Medicine at the University of Pennsylvania, Philadelphia, Pennsylvania, United States of America; 2 Key Laboratory of AIDS Immunology, Ministry of Health, The First Affiliated Hospital, China Medical University, Shenyang, Liaoning, People's Republic of China; 3 Howard Hughes Medical Institute and Department of Biochemistry and Biophysics, Perelman School of Medicine at the University of Pennsylvania, Philadelphia, Pennsylvania, United States of America; University of North Carolina at Chapel Hill, United States of America

## Abstract

The Epstein-Barr nuclear antigen 3C (EBNA3C), one of the essential latent antigens for Epstein-Barr virus (EBV)-induced immortalization of primary human B lymphocytes *in vitro*, has been implicated in regulating cell proliferation and anti-apoptosis via interaction with several cellular and viral factors. Gemin3 (also named DDX20 or DP103) is a member of DEAD RNA helicase family which exhibits diverse cellular functions including DNA transcription, recombination and repair, and RNA metabolism. Gemin3 was initially identified as a binding partner to EBNA2 and EBNA3C. However, the mechanism by which EBNA3C regulates Gemin3 function remains unclear. Here, we report that EBNA3C directly interacts with Gemin3 through its C-terminal domains. This interaction results in increased stability of Gemin3 and its accumulation in both B lymphoma cells and EBV transformed lymphoblastoid cell lines (LCLs). Moreover, EBNA3C promotes formation of a complex with p53 and Gemin3 which blocks the DNA-binding affinity of p53. Small hairpin RNA based knockdown of Gemin3 in B lymphoma or LCL cells remarkably attenuates the ability of EBNA3C to inhibit the transcription activity of p53 on its downstream genes p21 and Bax, as well as apoptosis. These findings provide the first evidence that Gemin3 may be a common target of oncogenic viruses for driving cell proliferation and anti-apoptotic activities.

## Author Summary

Gemin3 (DDX20 or DP103) is a member of the DEAD-box family of RNA helicases involved in various cellular processes including DNA transcription and RNA processing. The Epstein-Barr virus (EBV) encoded nuclear antigen 3C (EBNA3C) is essential for EBV-induced immortalization of primary human B-lymphocytes in vitro. In this study, we discovered that Gemin3 directly binds to the tumor suppressor p53, and acts as a negative regulator blocking p53 functions. Importantly, EBNA3C induces Gemin3 accumulation and enhances the formation of the complex of Gemin3 and p53 in EBV- transformed primary human B lymphocytes. Remarkably, inhibition of Gemin3 production leads to cell death of B lymphoma cells, particularly EBNA3C positive cells. This is the first evidence which shows that Gemin3 directly impairs p53 function in EBV positive cells, and that Gemin3 could be a potential target for EBV-associated cancer therapy.

## Introduction

Epstein-Barr virus (EBV) is the first identified human tumor virus which causes infectious mononucleosis [1],[2], and is linked several lymphoproliferative diseases [3], including Burkitt’s lymphoma [4], nasopharyngeal carcinoma [5], and Hodgkin’s disease [6]. EBV, a ubiquitous human γ-herpesvirus, infects more than 90% of the worldwide adult population. Moreover, AIDS patients or post-transplant patients whose immune system is suppressed have a high probability of developing EBV-associated lymphomas. In vitro, EBV can transform normal resting human B-cells to continuous proliferation of latently infected B cells resulting in lymphoblastoid cell lines (LCLs). Like other herpesvirus, the EBV life cycle exhibits both latent (non-productive) and lytic (productive) phases. Four types of latency programs are classified: Type I latency is mainly represented by Burkitt lymphoma (BL) cells; there are two EBER genes expressed, the BART transcripts, and EBNA1 (EBV nuclear antigen 1) [7]. Type II latency is most frequently seen in Hodgkin's lymphoma and nasopharyngeal carcinoma with three additional latent-membrane proteins, LMP-1, LMP-2A and LMP-2B expressed [8]. Latency III is seen predominantly in lymphoproliferative diseases developed in immunocompromised individuals and EBV-transformed lymphoblastoid cell lines [3] . In this group all six EBNAs, three LMPs and the two EBERs are expressed [7],[9]. Type IV latency is less strictly defined and is associated with infectious mononucleosis patients [8],[9]. Some infected individuals is associated with the tightly latent program (latency 0), in which latent gene expression is almost undetectable [9]. The essential mediators for EBV transformation of B lymphocytes and establishment of latency in vitro include EBNA2, EBNA3A, 3C and LMP1 proteins. Importantly, EBNA3C plays a complex regulatory role in the transcription of several viral and cellular genes. For example, EBNA3C targets the cellular transcription factor RBP-Jκ to antagonize EBNA2 mediated transactivation [10],[11], and cooperates with EBNA2 to activate the major viral LMP1 promoter via interaction with the cellular transcription factor, Spi-1/Spi-B [12]. EBNA3C also regulates chromatin remodeling by recruiting both histone acetylase and deacetylase activities [13]–[15]. Furthermore, EBNA3C modulates the transcription of cellular genes involved in cell migration and invasion by targeting the metastasis suppressor Nm23-H1 [16]. In addition to its transcriptional functions, it has been reported that EBNA3C has cell-cycle regulatory functions, presumably mediated by direct protein–protein interactions [13],[17]–[19]. EBNA3C also stabilizes c-Myc and interacts with Mdm2 in modulating p53 transcription and apoptotic activities [20]–[22].

Gemin3 was discovered as a binding partner with EBV latent antigens (EBNA2 and EBNA3C), and the survival motor neuron (SMN) protein [23],[24]. It consists of 825 amino acids with 9 conserved motifs including the ASP-Glu-Ala-Asp motifs (or DEAD box motif), and belongs to DExD/H RNA helicase family, which plays many roles in RNA metabolism including pre-mRNA splicing, ribosome biogenesis, RNA transport, translation initiation, and RNA decay [24]–[28]. Both EBNA2 and EBNA3C combine with Gemin3 and SMN,while EBNA2 cooperate with SMN in transactivation of the viral LMP1 promoter [24]–[26]. It has been shown that Gemin3 also interacts with and modulates a variety of cellular transcription factors including steroidogenic factor 1(SF-1) [29],[30], early growth response protein 2 (Egr2) [31], forkhead transcription factor FOXL2 [32] , and mitogen Ets repressor METS [33]. Although Gemin3 was shown to play a role in gene transcription regulation, the function of Gemin3 in cell proliferation remains largely unclear. Here we show that Gemin3 is stabilized by EBNA3C via protein-protein interaction and can play a role in cell proliferation through formation of a complex with p53 which results in blocking p53-mediated transcriptional activity and apoptosis pathway. Knockdown of Gemin3 by RNA interference dramatically increases apoptosis of EBV-infected LCLs.

## Results

### EBNA3C forms a complex and co-localizes with Gemin3 *in vivo*

Similar to a screen by Grundoff, et al [24], a previous yeast two-hybrid study showed that C-terminal domain of EBNA3C interacts with Gemin3. To confirm that these two molecules do associate in vivo, we performed co-immunoprecipitation assays to determine if EBNA3C forms a complex with Gemin3 in EBV transformed B lymphoma cell lines (LCL1 and LCL2). The B lymphoma cell line Ramos which lacks EBNA3C expression because it is EBV negative was used as a control. The results showed that endogenous Gemin3 was dramatically immunoprecipitated by anti-EBNA3C antibody, but not by control mouse serum (Figure 1A). The reverse immunoprecipitation with anti-Gemin3 antibody further confirmed that EBNA3C does form a complex with Gemin3 in vivo (Figure 1B). Since Gemin3 is initially identified as a binding protein of EBNA2 and EBNA3C, we wanted to determine if the EBNA3C complex with Gemin3 was independent of EBNA2 and performed similar coimmunoprecipitation assays again by using the EBV negative B lymphoma BJAB derived cell lines BJAB7 and BJAB10 with EBNA3C stable expression alone. The results showed that EBNA3C alone was sufficient to form a complex with Gemin3 in vivo (Figure 1C).

**Figure 1:** EBNA3C forms a complex with Gemin3 in EBV transformed cells. (A) and (B) Endogenous Gemin3 associates with EBNA3C. Twenty million of Ramos, LCL1, and LCL2 cells were individually lysed and subjected to immunoprecipitation (IP) with EBNA3C (A10) or Gemin3 (12H12) specific antibody. 5% of whole cell lysates (WCL) were loaded as input. Normal serum IgG was used for preclear (PC). Lysates and IP complexes were resolved by SDS-PAGE and subjected to western blotting (WB) with the indicated antibodies. (C) Exogenous EBNA3C associates with Gemin3. The EBNA3C stable expressing cells (BJAB7 and BJAB10) and parental BJAB cells were individually lysed and subjected to immunoprecipitation (IP) and western blotting as indicated.

To determine if the association of EBNA3C and Gemin3 occurs in the same cellular compartments in this scenario, we performed immunofluorescence assays by ectopically expressing FLAG-tagged EBNA3C and GFP-tagged Gemin3 in U2OS cells. The immunofluorescence results showed that although EBNA3C signals are shown as stippled, punctate dots with the exclusion of nuclei, and Gemin3 signal was displayed as intense staining of prominent but discrete foci in both nucleus and cytoplasm, and there were a number of positions where co-localization staining of EBNA3C with Gemin3 was evident (Figure 2A). To further visualize the interaction of these two proteins under physiological conditions, an EBV transformed cell line LCL1 was used. Endogenous EBNA3C and Gemin3 signals were evident with the co-localization pattern (Figure 2B), supporting the above data that these two proteins can associate in the same complex.

**Figure 2:** EBNA3C colocalizes with Gemin3. (A) Colocalization of exogenous E3C and Gemin3 in U2OS cells. Cells transfected with E3C-FLAG and GFP-Gemin3 were stained by using M2 antibody, followed by goat anti-mouse antibody conjugated to Alexa Fluor 594 (red). (B) Endogenous Gemin3 colocalizes with E3C in the EBV-transformed cell line LCL1. Endogenous Gemin3 and E3C were individually detected by using mouse anti-Gemin3 (12H12) and rabbit anti-E3C antibodies, followed by Goat anti-mouse antibody conjugated to Alexa Fluor 594 (red) and goat anti-rabbit antibody conjugated to Alexa Fluor 488 (green). Nuclei were counterstained by using DAPI (blue). The images were sequentially captured using an Olympus confocal microscope. All panels are representative pictures from similar repeat experiments. Enlarged sections are shown at the bottom. Arrows show the colocalization of E3C and Gemin3.

### EBNA3C interacts with Gemin3 through its C-terminal domains

To define which domain of EBNA3C interacts with Gemin3, we co-transfected HEK293 cells with expression constructs for GFP-tagged Gemin3 and FLAG-tagged full-length (residues 1 to 992) or a series of truncated mutant of EBNA3C (1–365, 366–620, or 621–992), and performed coimmunoprecipitation assays with GFP or FLAG antibodies. Consistently, the results showed that coimmunoprecipitation targeting Gemin3 or EBNA3C, always results in Gemin3 co-immunoprecipitating with both the full-length and C-terminal domain of EBNA3C with relatively high affinity (Figure 3A and B). To further determine if the C-terminal domain of EBNA3C alone is sufficient to bind with Gemin3, we performed GST pulldown assays by in vitro-translating the full length and truncated mutants of EBNA3C followed by co-incubation with bacterially expressed GST-Gemin3 protein. The results showed that the C-terminal domain (621–992) of EBNA3C directly interacted with Gemin3 (Figure 3C). Similarly, using in vitro-translated Gemin3 coincubated with different bacterially expressed GST-EBNA3C (1–365, 366–581, 582–792, and 900–992), we further found that the C-terminal amino acids 621 to 792, a smaller region than previously identified by yeast two-hybrid analysis (534–778aa, [24]) of EBNA3C was critical for binding to Gemin3 in vitro (Figure 3D and F). To determine the domain of Gemin3 responsible for interacting with EBNA3C, we generated three truncated mutants of GST-Gemin3 (residues 1–272, 307–547 and 546–825) and performed GST pulldown assays with in vitro-translated full-length EBNA3C. The result showed that Gemin3 bound with EBNA3C via its C-terminal domain (Figure 3E and F), supporting the previously identified data by yeast two-hybrid analysis [24], and further narrows the interacting domain.

**Figure 3:** EBNA3C and Gemin3 interact through their C-terminal domains. (A) and (B) Gemin3 associates with the C-terminal domain of EBNA3C. Twenty million of HEK 293 cells were cotransfected with plasmids expressing GFP-tagged Gemin3 and Flag-tagged either full-length or the truncated mutants of EBNA3C. At 36 h post-transfection, cells were harvested and subjected to immunoprecipitation using anti-FLAG (M2) or GFP antibodies followed by western blotting with GFP or M2 antibody. 5% of whole cell lysates (WCL) were used as input. The membrane was stripped and reblotted with M2 or GFP antibody. (C) Gemin3 binds to C-terminal domain of E3C in vitro. The ^35^S-radiolabeled in vitro-translated proteins of E3C truncated mutants were precleared with GST bead, followed by incubation with GST or GST-Gemin3 beads. The bound protein mixtures were resolved by appropriate SDS-PAGE, and autography. 5% of in vitro translated protein is used as input. The quantification of relative amount of bound protein (RBU) was shown at the bottom. (D) The ^35^S-radiolabeled in vitro-translated protein full-length Gemin3 was pulled down by truncated mutants of EBNA3C fusion with GST (GST-E3C 1–365, 366–581,582–792, and 900–992). Coomassie blue staining of purified GST-EBNA3C truncated proteins is shown at the bottom panel. (E) E3C binds to C-terminal domain of Gemin3 in vitro. The ^35^S-radiolabeled in vitro-translated protein full-length EBNA3C was pulled down by truncated mutants of Gemin3 fusion with GST (GST-Gemin3 1–272, 307–547, and 546–825). Coomassie blue staining of purified GST-Gemin3 truncated proteins is shown at the bottom. (F) Schematics illustrate different structural domains of E3C and Gemin3. The respective binding domain(s) of two proteins are indicated by bold.

### EBNA3C enhances the protein stability and production of Gemin3

To determine if EBNA3C plays a role on the production of Gemin3, we tested endogenous Gemin3 protein levels in EBNA3C stable expressing cell lines (BJAB7 and BJAB10) and parental BJAB cells, as well as EBV negative Ramos cells. Interestingly, the results showed that EBNA3C greatly induced the production of Gemin3 in BJAB cells (Figure 4A). To verify if whole EBV latent infection with EBNA3C expression also has the same effect on Gemin3 production, we did a western blot to detect Gemin3 protein levels in both PBMC and two EBV-infected derived LCL cell lines. Consistent with EBNA3C expression alone, the results showed that Gemin3 protein levels were significantly increased by EBV infection (Figure 4B). The results of Gemin3 protein levels in EBNA3C-knockdown BJAB10 and LCL cells were consistently much lower than in the control cells (Figure 4C), further suggesting that EBNA3C is required for maintenance of Gemin3 levels. To determine if the increased production of Gemin3 is due to post-translational regulation by EBNA3C, we co-expressed exogenous EBNA3C-FLAG with GFP-Gemin3 or GFP control vector into Saos-2 cells and determined the protein levels of GFP-Gemin3 and GFP. The results showed that the production of GFP-Gemin3 but not GFP was enhanced by EBNA3C in a dose-dependent manner (Figure 4D, left and middle panels), indicating that the interaction of EBNA3C with Gemin3 is important for Gemin3 accumulation. To this end, we carried out similar experiments by using an EBNA3C mutant lacking Gemin3-interacting domain, and found that deletion of the Gemin3-interacting domain efficiently abolished the effect of EBNA3C on Gemin3 production (Figure 4D, left and right panels). To further confirm that EBNA3C-induced Gemin3 levels were due to enhanced Gemin3 protein stability, we performed the protein stability assays for Gemin3 by treating BJAB (EBNA3C negative) and BJAB10 (EBNA3C positive) cells with cycloheximide (a protein translation inhibitor). The results showed that the stability of Gemin3 was dramatically enhanced in the presence of EBNA3C compared to cells without EBNA3C (Figure 4E).

**Figure 4:** EBNA3C enhances the protein stability of Gemin3. (A) and (B) E3C increases the protein production of endogenous Gemin3. Ten million of EBV negative cells (Ramos, BJAB and PBMC), EBNA3C- expressing cells (BJAB7 and BJAB10), and EBV-transformed cells (LCL1 and LCL2) were lysed and subjected to western blot with indicated antibodies. The data show that the protein level of Gemin3 in the EBNA3C or EBV positive cells was significantly upregulated. (C) The protein level of Gemin3 is decreased in BJAB10 and LCL1 cells with EBNA3C stable knockdown. BJAB10 and LCL1 cells with Lentivirus-delivered GFP labeled shRNA against EBNA3C (shE3C) or scramble control (shCtrl) were showed on the left panel. The protein levels of E3C and Gemin3 are detected by western blotting with indicated antibodies. GAPDH immunoblotting was used as the loading control. The relative quantitation of Gemin3 and E3C protein levels are normalized by GAPDH. (D) E3C increases the protein level of exogenous Gemin3. Saos-2 cells were transfected GFP-Gemin3 or GFP with increasing amounts of full length (FL) EBNA3C-FLAG or its C-terminal deleted mutant (ΔC). The transiently transfected cells were harvested at 36 h post-transfection, the protein levels of exogenous GFP-Gemin3 and GFP were detected by western blotting with GFP antibody. The relative quantitation of GFP-Gemin3 or GFP is shown in the middle panel. (E) EBNA3C enhances the protein stability of Gemin3. The cell lysates of BJAB or BJAB10 cells treated with cycloheximide (CHX, 100 µg/ml) for 0, 2, 4 and 6 hours were subjected to immunoblotting as indicated. GAPDH immunoblotting was used as the loading control. The relative quantitation of Gemin3 is shown in the middle panel.

### Gemin3 interacts with p53 and contributes to EBNA3C-mediated inhibition of p53 transcriptional activity

Our previous studies showed that EBNA3C blocks p53-mediated transcriptional as well as apoptotic activity [22],[34]. Gemin3 plays an essential role in cell survival and can function as a transcriptional repressor through interaction with a number of transcriptional factors [35],[36]. Therefore, we hypothesized that EBNA3C enhanced Gemin3 levels may be due to its interaction with p53 and in turn repress the transcriptional activity of p53. To this end, we first asked if Gemin3 can directly bind to p53 in vitro. Using in vitro-translated Gemin3, we incubated it with bacterially expressed GST or GST-p53 protein. We found that Gemin3 strongly bound to p53 but not the GST control (Figure 5A, lane 2 and 3). Using different truncation mutants of p53 fusion with GST, we found that the DNA-binding domain (amino acids 100–300) of p53 is critical for interaction with Gemin3 (Figure 5A, lane 4 to 6). To define the binding site of Gemin3 with p53, we utilized full length and truncated mutants of Gemin3 fusion with GST to incubate with in vitro-translated p53. The results showed that the C-terminal domain (amino acids 546–825) alone of Gemin3 presents similar strong binding with p53 as full length Gemin3 (Figure 5B). This further confirms that Gemin3 can directly interact with p53. To test if endogenous p53 interacts with Gemin3 in cells and whether this interaction is impaired by EBNA3C, we performed immunoprecipitation assays with anti-p53 antibody followed by western blotting with Gemin3 antibody individually from cell lysates of BJAB, BJAB10 and LCL1 cells. The results showed that Gemin3 and p53 do form a complex in EBV negative BJAB cells, and that the association of p53 with Gemin3 was greatly enhanced by 2.2 fold in EBNA3C-expressing BJAB10 cells and 5.2 fold in LCL1 cells when compared to that in the EBV negative BJAB cells (Figure 5C, bottom panel). Since Gemin3 bound to the DNA-binding domain of p53, we wanted to know if Gemin3 blocks sequence specific DNA-binding ability of p53, and so performed chromatin immunoprecipitation assays with exogenous p53 alone or p53 and Gemin3 in the presence and absence of p53-responsive DNA element (p53-RE). As shown in the Figure 5D, Gemin3 dramatically reduced the ability of p53 to bind to the p53-responsive DNA element. To further confirm the consequence of Gemin3 blocking DNA-binding ability of p53 and argue the possibility that Gemin3 can directly bind to DNA probe, we also performed reporter assays by co-expressing exogenous HA-p53 with increasing doses of GFP-tagged Gemin3 in the presence of 13 copies of p53-binding sites driven luciferase reporter into p53-null Saos-2 cells. The results showed that Gemin3 diminished p53-mediated transcriptional activity in a dose-dependent manner (Figure 5E). The expression levels of Gemin3, p53, and GAPDH as a loading control, were also analyzed by western blotting (Figure 5E, bottom panels). To answer if EBNA3C-mediated inhibition of p53 transcriptional activity is dependent on Gemin3 accumulation, we performed similar reporter assays by co-expressing p53 with or without EBNA3C in the presence of specific Gemin3 shRNA (shG3) or non-specific control shRNA (shCtrl). Strikingly, the results showed that EBNA3C-mediated inhibition of p53 transcriptional activity is dramatically reversed once Gemin3 is knocked down (Figure 5F, compare lane 3 with 6). This suggests that Gemin3 is important for EBNA3C-mediated inhibition of p53 function.

**Figure 5:** Gemin3 interacts with p53 and contributes to EBNA3C-mediated inhibition of p53 transcriptional activity. (A) Gemin3 binds with DNA-binding domain of p53 in vitro. ^35^S-radiolabeled Gemin3 was in-vitro translated and incubated with bacterially purified GST, GST fusion with full length (1–393) or truncated mutants of p53 (1–83, 100–300, and 300–393). The pull-down complexes were resolved by appropriate SDS-PAGE and autography. The amount of bound protein was quantified with ImageQuant software. Coomassie blue staining of purified GST protein is shown in the middle panel. Schematic illustrates the binding domains of p53 with Gemin3 and EBNA3C. (B) C-terminal domain of Gemin3 binds with p53 in vitro. ^35^S-radiolabeled p53 was in vitro translated and incubated with bacterially purified GST control, full length GST-Gemin3 (1–825) or its truncations (1–272, 307–547, and 546–825). The GST pull down assay was analyzed as the described above. (C) EBNA3C increases the interaction of p53 with Gemin3. Twenty million of BJAB, BJAB10 and LCL1 cells were individually harvested, lysed and subjected to immunoprecipitation (IP) with p53 specific antibody and subsequently western blotted with Gemin3 or p53 antibody. The relative quantitation of Gemin3 complex with p53 was calculated by IP compared with input and shown in bottom panel. (D) Gemin3 reduces DNA-binding affinity of p53. Saos-2 cells were co-transfected HA-p53 with or without GFP-Gemin3 in the presence of p53-RE-Luc containing 13 copies of p53-binding sties or pGL3-basic vector alone. Chromatin immunoprecipitation assays were performed with anti-HA or normal lgG antibodies control. The DNA binding ability of p53 was detected by standard (upper) and quantitative real-time (lower) PCR with primers targeting ampicilin gene of pGL3 plasmid. (E) Gemin3 inhibits the transcriptional activity of p53 in the luciferase reporter assay. Saos-2 cells were co-transfected with 3 µg of the pGL3-p53-RE-Luc, 10 µg HA-p53 in the presence of either vector control or increasing amounts of GFP-Gemin3 (5 µg and 10 µg). Each transfection was performed in triplicate. Error bars indicated standard variations. Bottoms panels show the protein levels detected by western blotting analysis with the indicated antibodies. GAPDH was used as a control for equal loading. The relative luciferase unit (RLU) is showed by normalization with vector alone. (F) Gemin3 knockdown reduces E3C-mediated inhibition of p53 transcriptional activity in the luciferase reporter assays. Saos-2 cells with stable Gemin3 knockdown (shG3) or control (shCtrl) were individually co-transfected p53-RE-Luc with HA-p53, HA-p53 and E3C-FLAG or vector alone. The western blotting data of each protein is shown at the bottom panel. The relative luciferase unit (RLU) is showed by normalization with vector alone. Plasmid expressing RFP was used for normalized transfection efficiency.

### Gemin3 knockdown attenuates EBNA3C-mediated inhibition of p53-induced apoptosis

Studies in our lab have shown that EBNA3C is able to inhibit p53-induced apoptosis in p53-null Saos2 cells [22],[34]. To further confirm the significance of Gemin3 on EBNA3C-mediated inhibition of p53 function, we verified whether or not Gemin3 knockdown affects EBNA3C-mediated inhibition of p53-induced apoptosis by using colony formation assays. The results showed that coexpression of EBNA3C with p53 markedly increased the colony formation of Saos-2 cell compared to that produced by p53 alone (Figure 6A, left panel). In contrast, although less colony formation was produced in the vector alone with the Gemin3 knockdown (shG3) compared to that with the control knockdown (shCtrl) (Figure 6A, top panel), the colony formation of p53 co-expressed with EBNA3C was significantly inhibited in Gemin3 knockdown cells (Figure 6A). Thus, these data revealed a role for EBNA3C in upregulation of Gemin3 for anti-apoptosis and promotes cell proliferation.

**Figure 6:** Gemin3 knockdown attenuates EBNA3C-mediated inhibition of p53-induced apoptosis. (A) Saos-2 (p53^−/−^) cells were electroporated with different combinations of expression plasmids for HA-p53, EBNA3C-FLAG or vector alone in the presence of small hairpin RNA against Gemin3 (shG3) or control (shCtrl) as indicated. 2×10^3^ transfected cells were cultured in the selection medium (DMEM supplemented with 100 mg/ml G418). After a 2-week selection, cells were fixed on the plates with 4% formaldehyde and stained with 0.1% crystal violet. The area of colonies (pixels) in each dish was calculated by LiCor Odyssey. The number represents the averages of data from two independent experiments. Plasmid expressing RFP was used for normalized transfection efficiency. (B) Western blots showing the protein level of Gemin3 in the lentivirus-mediated Gemin3 or control knockdown cell lines. GAPDH was used as the loading control. (C) Gemin3 knockdown increases apoptosis of EBV negative cells (Ramos and BJAB), EBNA3C positive cells (BJAB7 and BJAB10), and EBV transformed cells (LCL1). Cells were harvested after a 12-h serum starvation and fixed. Levels of cells undergoing apoptosis (sub-G1 phase) in individual PI-stained samples were detected by flow cytometry, and the data were analyzed by FlowJo software. The bar diagram shown at the bottom panel represents the mean of three independent experiments and the results of comparing with each control knockdown sample. (D) Quantitative real-time PCR analysis showed that p53, p21 and Bax genes were upregulated in the Gemin3 knockdown cells. Total RNA was individually isolated from the Gemin3 (shG3) or control (shCtrl) knockdown cells with 12-h serum starvation treatment. A 2 µg total RNA was used to synthesis cDNA. Error bars show standard deviations.

To further prove that Gemin3 plays an important role in cell proliferation, we performed apoptosis assays using B lymphoma cells or LCLs with or without lentivirus-mediated Gemin3 knockdown. Gemin3 expression was significantly knocked down in the EBV negative B lymphoma cell lines Ramos and BJAB, EBV transformed B cell line LCL1 as well as EBNA3C stably expressing BJAB cell lines BJAB7 and BJAB10 (Figure 6B). The results of apoptotic assays showed that Gemin3 knockdown cells had a dramatic increase in apoptosis compared to the control knockdown cells (Figure 6C). Furthermore, Gemin3 knockdown in EBV or EBNA3C positive cells showed significantly higher levels of apoptosis than that in EBV or EBNA3C negative cells (Figure 6C, bottom panel). Consistently, the quantitative PCR analysis showed that the transcriptional levels of p53 downstream genes including p21, Bax and p53 were enhanced when Gemin3 was knocked down in EBNA3C positive cells and were remarkably higher than that in EBNA3C negative cells (Figure 6D). Therefore, Gemin3 plays a critical role in cell proliferation in EBNA3C positive cells.

## Discussion

Emerging evidence have indicated that Gemin3 is an essential gene for embryonic development and survival from mammal to Drosophila [23],[37]. Gemin3 (DP103/DDX20) was originally discovered in a screen for cellular factors that bind to EBNA2 and EBNA3C using the yeast two-hybrid system [24]. Gemin3 was shown to be involved in EBNA2-mediated transactivation and transformation, and a deletion mutant of EBNA2 lacking the Gemin3-binding site severely impeded LMP1 transactivation and viral transformation [26]. However, there was no previous report on the functional effect of EBNA3C on Gemin3. Our yeast two-hybrid screen showed that Gemin3 strongly interacted with EBNA3C and this was identified with high frequency in positive yeast clones when the C-terminal domain of EBNA3C was used as bait (data not shown). We now confirm that Gemin3 directly binds to EBNA3C in vitro and in vivo, and this interaction led to increased Gemin3 protein stability and its accumulation in B lymphoma cells and EBV-transformed lymphoblastoid cell lines. Furthermore, EBNA3C promoted the formation of a complex with p53 and Gemin3 in vivo which was important for blocking p53-mediated transcriptional activity and apoptosis. Inhibition of Gemin3 expression dramatically abolished EBNA3C-mediated inhibition of p53-induced apoptosis (Figure 7). The emerging evidence showing Gemin3 as a DEAD-box RNA helicase that plays a role in carcinogenesis, will inspire us to develop efficient helicase inhibitors as a potential target for anti-cancer in the future.

**Figure 7:** A schematic model depicting the Gemin3-mediated transcriptional regulation of p53 by EBNA3C in the EBV latently infected cells. *Left panel*, in response to genotoxic stress, p53 achieves its anti-proliferative properties through its function as a DNA-binding transcriptional activator, and induce expression of downstream target genes (including p21 and BAX) for cell-cycle arrest and apoptosis. *Right panel*, in the EBV latency III cells, EBNA3C not only stabilizes Gemin3 through the interaction of their C-terminal domains and but also enhances a stable complex of Gemin3 with p53 for blocking p53-mediated transcriptional activity and cell apoptosis. Gemin3 knockdown (siRNA) increases the sensitivity of the EBNA3C-expressing cells to stress-induced apoptosis. p53-RE, p53 responsive element.

Gemin3 is also an integral component of the SMN complex, which plays an essential role in the production of spliceosomal small nuclear ribonucleoproteins (snRNPs) [38], regulation of DNA transcription [30], pre-mRNA splicing [37], and axonal RNA transport [39]. In addition to interaction with Gemin3, EBNA3C also has been shown to associate with SMN [25]. This further supports the notion that EBNA3C targets the SMN complex and can impair the function of each component including Gemin3 in the SMN complex. Here, we demonstrate a novel function of Gemin3 as a regulator that suppresses p53-mediated transcriptional activity and apoptosis. Interestingly, SMN was also shown to interact with p53 [40]. Therefore, our results showing that knockdown of Gemin3 sufficiently rescues p53, suggest that Gemin3 could be a critical member of the SMN complex to suppress p53 function. This provides an explanation as to why EBNA3C promotes complex formation of p53 and Gemin3 through enhancing Gemin3 protein stability.

The N-terminal domain of Gemin3 contains the conserved helicase motifs, while the non-conserved C-terminal domain can interact with a variety of cellular and viral factors. In this study, we found that Gemin3 binds with both EBNA3C and p53 through the same region (amino acid 548 to 825) of its C-terminal domain. Considering that EBNA3C individually binds to p53 and Gemin3 through its N-terminal and C-terminal domains. There is a strong possibility for EBNA3C to act as an adaptor to promote Gemin3 interaction with p53. This also may provide an explanation as to why the levels of p53 in complex with Gemin3 are dramatically enhanced in the presence of EBNA3C.

Although it has been shown that Gemin3 plays a diverse roles on repressing gene transcription [30], the mechanism of Gemin3-mediated transcriptional repression is not fully clear. One of the potential mechanisms could be through recruitment of specific transcription co-repressors. For examples, Gemin3 interacts with METS to repress Ets by assembling a complex of N-CoR, Sin3A, HDAC-2, and HDAC-5 [30],[33],[41]. Gemin3 was also found to form a complex with METS (mitogenic Ets transcriptional suppressor)/PE1 or ERF (Ets2 repressor factor) controlling cellular proliferation and differentiation through recruitment of HDAC2 and HDAC5 [42]. It also interacts with and represses the transcriptional activity of Egr2/Krox-20 which is dependent in part on HDAC recruitment [31]. Gemin3 also interacts with the transcriptional factor FOXL2 important for inducing apoptosis [32]. However, our study showed that Gemin3 reduces p53 transcriptional activity and now provides another potential mechanism through which Gemin3 can sequester a transactivation cofactor or may disrupt a transcriptionally active nucleic acid-protein complex.

Previous studies in our lab indicated that EBNA3C targets multiple factors to deregulate the p53 pathway and so drive cell proliferation. For example, EBNA3C has a unique activity of ubiquitylation and de-ubiquitylation [17],[18],[21], and also suppresses p53 function through formation of a complex with Mdm2 [21]. More recently, our lab also showed that EBNA3C directly competes with two p53-associated growth inhibitors ING4 and ING5 for attenuating p53 function [34]. Despite current studies which convincingly showed that EBNA3C inhibit p53 function, it is still unknown as to why the protein level of p53 is not affected in EBV-transformed LCLs or in B lymphoma expressing EBNA3C [43]–[46]. Here, our study further addresses a potential mechanism that EBNA3C can block p53 function through upregulating Gemin3 protein levels and so promoting the formation of a complex of p53 with Gemin3. This is distinctly different from the strategy used by KSHV encoded LANA where p53 ubiquitylation is induced and results in its degradation [47]. In summary, this study provides initial evidence that Gemin3 can directly interact with p53 through its DNA-binding domain and in turn inhibits its activities. This pathway is essentially targeted by EBNA3C in EBV-transformed lymphoblastoid cells.

## Materials and Methods

### DNA constructs and antibodies

pA3F-EBNA3C constructs expressing either full-length EBNA3C or different truncated versions of EBNA3C 1–365, 366–620, and 621–992 with a Flag tag at the carboxy-terminal end and Glutathione S-transferase (GST)-EBNA3C truncation mutation were described previously [20]. Constructs expressing green fluorescent protein (GFP)-tagged Gemin3 was prepared by cloning PCR-amplified fragments into pEGFP-C1 vector (BD Biosciences Clontech) at *EcoR*I and *Sal*I restriction sites. The plasmid pGL3-p53-RE contains 13 copies of p53-binding site at the upstream of firefly luciferase gene was constructed by *EcoR*V insertion of p53-binding sequences into the pGL-3 luciferase reporter plasmid (Kindly provided by Wafik S. EI-Deiry at University of Pennsylvania, Philadelphia, Pennsylvania). pGEX-p53 expresses an N-terminal glutathione S-transferase (GST)-p53 fusion protein was derived from pGEX-2T (Amersham Pharmacia, Inc, Piscataway, NJ) by insertion of human p53 cDNA (A gift from Gary J Nabel, National Institutes of Health, Bethesda, MD) at the *Bam*H1 and *Eco*R1 sites. pcDNA-HA-p53 was generated by cloning PCR-amplified p53 cDNA using pGEX-p53 as a template into the pcDNA3-HA vector at *Eco*R1 and *Not*1 sites. GST-p53 truncation mutants were constructed by insertion of PCR fragments into the pGEX-5x-1 backbone (gift from Shelley L Berger, The Wistar Institute, Philadelphia, PA). Plasmid expressing GST-Gemin3 was kindly provided by Dr. Gideon Dreyfuss (Howard Hughes Medical Institute Investigator at University of Pennsylvania Perelman School of Medicine) and described previously [23]. GST-Gemin3 truncation mutants GST-Gemin3 1–272 was constructed by insertion of PCR fragments into pGEX-2TK derivative vector at *Kpn*1 and *Eco*R1 sites, GST-Gemin3 307–547 and GST-Gemin3 546–825 into pGEX-2TK vector *Bam*H1 and *Eco*R1 sites. All constructs and mutations were verified by DNA sequencing.

Mouse monoclonal anti-Gemin3 (12H12) was kindly provided by Dr. Gideon Dreyfuss (Howard Hughes Medical Institute Investigator at University of Pennsylvania School of Medicine). The monoclonal antibodies mouse anti-myc (9E10) and anti-EBNA3C (A10) were prepared from the respective hybridoma cultures. Mouse monoclonal antibody anti-FLAG epitope (M2) was purchased from Sigma-Aldrich Corp. (St. Louis, MO). Mouse monoclonal antibody reactive to p53 (DO-1) and GFP (F56-BA1) were purchased from Santa Cruz Biotechnology, Inc. (Santa Cruz, CA).

### Cell culture and transfection

Human embryonic kidney cells transformed with sheared adenovirus type 5 DNA HEK293 cell line and p53-null cell line SaoS-2 were obtained from Jon Aster (Brigham and Woman’s Hospital, Boston, MA) [48]. U2OS is also a human osteosarcoma cell line [49]. EBV negative Burkitt’s lymphoma cell lines BJAB and Ramos were provided by Elliott Kieff (Brigham and Woman’s Hospital, Boston, MA) [50]. LCL1 and LCL2 are in vitro-transformed EBV positive cell lines. BJAB cells expressing EBNA3C (BJAB7 and BJAB10) were generated previously by transfecting with pZipneo eukaryotic expression vector with EBNA3C cDNA followed by neomycin selection [51]. HEK 293, U2OS and Saos-2 cells were grown in Dulbecco's modified Eagle's medium (purchased from HyClone, Logan, UT) supplemented with 10% fetal bovine serum, 50 U/ml penicillin, 50 µg/ml streptomycin, and 2 mM L-glutamine. BJAB, Ramos and the EBV-positive cell lines were maintained in RPMI 1640 medium (HyClone, Logan, UT) supplemented as described for Dulbecco's modified Eagle's medium above. All cultures were incubated at 37°C in a humidified environment supplemented with 5% CO2. Cells were transfected by electroporation with a Bio-Rad Gene Pulser II electroporator. Briefly, 15×10^6^ cells harvested in exponential phase were collected, washed in phosphate-buffered saline (PBS), and resuspended in 400 µl of the appropriate medium containing DNA for transfection [52]. Resuspended cells were transferred to a 0.4-cm-gap cuvette, and electroporation was performed at 975 µF, 210 V for HEK293 and Saos-2 cells. Transfected cells were transferred to a 100-mm petri dish containing 10 ml of complete medium and incubated at 37°C.

### Immunoprecipitation and Western blotting

Transfected cells were harvested, washed with ice-cold PBS, and lysed in 0.5 ml ice-cold radioimmunoprecipitation (RIPA) buffer (1% Nonidet P-40 [NP-40], 10 mM Tris [pH 7.5], 2 mM EDTA, 150 mM NaCl), supplemented with protease inhibitors (1 mM phenylmethylsulfonyl fluoride, 1 µg/ml aprotinin, 1 µg/ml pepstatin, and 1 µg/ml leupeptin). Cell debris was removed by centrifugation at 21,000×g (10 min and 4°C), and the supernatant was transferred to a fresh microcentrifuge tube. Lysates were then precleared by end-over-end rotation with normal mouse serum and 30 µl of a 1∶1 mixture of Protein A-Protein G-conjugated Sepharose beads (1 h, 4°C). Beads were spun out, and supernatant was transferred to a fresh microcentrifuge tube and approximately 5% of the lysate was saved for input control. The protein of interest was captured by rotating the remaining lysate with 1 µg of appropriate antibody overnight at 4°C. Immune complexes were captured with 30 µl of a 1∶1 mixture of Protein A and Protein G Sepharose beads, pelleted, and washed five times with ice-cold RIPA buffer. For Western blot assays, input lysates and immunoprecipitated (IP) complexes were boiled in Laemmli buffer [53], fractionated by SDS-PAGE, and transferred to a 0.45 µm nitrocellulose membrane. The membranes were then probed with appropriate antibodies followed by incubation with appropriate infrared-tagged secondary antibodies and viewed on an Odyssey imager (LiCor Inc., Lincoln, NE).

### Purification of GST fusion proteins

Escherichia coli BL21 (DE3) cells were transformed with the plasmid constructs for each GST fusion protein. Single colonies were picked and grown overnight in 3 ml of Luria broth supplemented with 100 µg/ml ampicillin. One milliliter of the overnight culture was used to inoculate a 500 ml culture. The larger culture was incubated until the optical density at 600 nm was approximately 0.6, at which point it was induced with 1 mM isopropyl-β-D-thiogalactopyranoside (IPTG) for 12 h at 30°C . The bacteria were pelleted, washed once with STE buffer (100 mM NaCl, 10 mM Tris, and 1 mM EDTA, pH 7.5), resuspended in 3 ml NETN buffer (0.5% NP-40, 100 mM NaCl, 20 mM Tris, 1 mM EDTA, pH 8.0), supplemented with protease inhibitors, and incubated on ice for 15 min. A volume of 150 µl of 1 M dithiothreitol (DTT) and 1.8 ml of a 10% solution of Sarkosyl in STE buffer was added, and the suspension was sonicated (for 3 min on ice) to solubilize the proteins. The lysates were centrifuged (12,000×g, 10 min, 4°C) to separate the unsolubilized fraction. The clear supernatant was transferred to a fresh tube, to which 3 ml of 10% Triton X-100 in STE buffer and 200 µl of Glutathione-Sepharose beads were added. The tube was rotated overnight at 4°C, after which the purified protein bound to Glutathione was collected by centrifugation (2 min, 600×g, 4°C) and washed five times with NETN buffer supplemented with protease inhibitors. The level of purification was determined by SDS-PAGE, and purified proteins were stored at 4°C.

### GST pull-down assays

For pull-down assays from cell lysates, lysates were prepared in RIPA buffer (0.5% NP-40, 10 mM Tris [pH 7.5], 2 mM EDTA, 150 mM NaCl, supplemented with protease inhibitors). Lysates were precleared and then rotated with either GST control or the appropriate GST fusion protein bound to Glutathione-Sepharose beads. For in vitro binding experiments, GST fusion proteins were incubated with ^35^S-labeled in vitro-translated protein in binding buffer (1×PBS, 0.1% NP-40, 0.5 mM DTT, 10% glycerol, supplemented with protease inhibitors). In vitro translation was performed with the T7-TNT Quick Coupled transcription-translation system (Promega Inc., Madison, WI) according to the manufacturer's instructions.

### Immunofluorescence

To check the co-localization of ectopically expressed GFP-Gemin3 and Flag-EBNA3C in the cells, we used Lipofectamine 2000 (Invitrogen, Carlsbad, CA) to transfect U2OS cells with the plasmids then cultured on coverslips. At 36 h posttransfection, cells were fixed using 3% paraformaldelhyde with 0.1% Triton X-100 for 20 min at room temperature. We used LCL1 cells to examine the co-localization of endogenous Gemin3 with EBNA3C, appropriate LCL1 cells were added onto slides and fixed using the same method after culture 5 h. Fixed cells were washed with PBS and subsequently blocked in 1% BSA for 10 min. Gemin3 was detected using mouse monoclonal antibody (12H12). Endogenous EBNA3C was detected using EBNA3C-reactive rabbit polyclonal antibody (1∶150 dilution); Flag-tagged EBNA3C was detected using M2 antibody (1∶1,000 dilution; Santa Cruz Biotechnology, Inc., Santa Cruz, CA). Primary antibodies were incubated with the cells for 60 min at the room temperature. Cells were washed three times with PBS and exposed to secondary antibodies. Goat anti-mouse antibody conjugated to Alexa Fluor 594 to detect Gemin3 and goat anti-rabbit antibody conjugated to Alexa Fluor 488 to detect EBNA3C were respectively used for LCL1 cells, and Goat anti-mouse antibody conjugated to Alexa Fluor 594 to detect FLAG-EBNA3C was used for U2OS cells. Secondary antibodies were diluted in blocking buffer at 1∶1,000 and incubated for 1 h at RT, followed by three washes with blocking buffer. The last wash contained 4′, 6′-diamidino-2-phenylindole (DAPI; Promega, Madison, WI) to counterstain the nuclei. The slides were examined using Olympus confocal microscopy and the images were analyzed with a Fluoview FV300 (Olympus, Melville, NY) software.

### Luciferase reporter assay

Twelve million Saos-2 cells were co-transfected by using a Bio-Rad electroporater (Bio-Rad Laboratories, Inc., Hercules, CA) with different combination of pGL3-p53-RE, pcDNA-HA-p53, pA3F-EBNA3C and GFP-Gemin3. At 24 h post-transfection, cells were harvested, washed in PBS, and lysed by cell lysis buffer (BioVision, Inc., Mountain View, CA). Forty microliters of cell lysate was used for the reporter assay, using an LMaxII384 luminometer (Molecular Devices, Inc., Sunnyvale, CA). A portion of the cell lysate was used for Western blotting. Transferred proteins were detected with Odyssey infrared scanning technology (LI-COR, Inc., Lincoln, NE), using Alexa Fluor 680 and Alexa Fluor 800 (Molecular Probes, Carlsbad, CA, and Rockland, Gilbertsville, PA, respectively). All the transfections were performed multiple times, and the results shown represent the means of the data from three independent experiments.

### Lentiviral-mediated gene silencing

For the lentivirus-mediated knockdown of EBNA3C or Gemin3, the EBNA3C shRNA sequence (CCAUAUACCGCAAGGAAUA) or Gemin3 shRNA (ACUCCCCAGUGAGACCAUU) was respectively inserted into pGIPZ vector according to the manufacture’s instructions (Open Biosystem, Inc, Huntsville, AL), the vector expressing EBNA3C or Gemin3 small hairpin RNA is abbreviated as shE3C or shG3, respectively. A 21-mer oligonucleotide (UCUCGCUUGGGCGAGAGUAAG) that had no significant homology to any known human mRNA in the databases was cloned in the same vector and used as control. Control shRNA is hereinafter abbreviated as shCtrl.

Lentiviruses were produced by transient transfection into HEK 293T cells as previously described with the following modifications [54]. A total of 2×10^6^ 293T cells were seeded in 10-cm-diameter dishes in DMEM (HyClone, Logan, UT) supplemented with 10% FBS and cultured for 24 h prior to transfection. A total 20 µg of plasmid DNA was used for the transfection of each dish, including 1.5 µg of envelope plasmid pCMV-VSV-G (catalog no. 8454; Addgene, Inc., Cambridge, MA), 3 µg of packaging plasmid pRSV-REV (catalog no. 12251 Addgene, Inc., Cambridge, MA), 5 µg of packaging plasmid pMDLg/Prre (catalog no. 12251 Addgene, Inc., Cambridge, MA), and 10.5 µg of lentiviral vector plasmid. The precipitation was formed by adding the plasmids to a final volume of 438 µl of H_2_0 and 62 µl of 2 M CaCl_2_, mixing well, adding 500 µl of 2×HEPES-buffered saline, and then incubating at room temperature for 30 min. Chloroquine was added to the 10 ml of plated media with a final concentration of 25 µM at 5 minutes prior to transfection. The medium was replaced after 12 h with DMEM supplemented with 10% FBS and 10 mM HEPES, and 10 mM sodium butyrate. The medium was replaced again 10 hours later using DMEM supplemented with 10% FBS and 10 mM HEPES. The conditioned medium was collected four times at 12 h interval, filtered through 0.45 µm pore-size cellulose acetate filters, and stored on ice. The virus was concentrated by spinning at 70,000×g for 2.5 h. The concentrated virus was resuspended in RPMI then used to infect 10^6^ cells in the presence of 20 µM/ml Polybrene. After 72 h, add puromycin to final concentration of 2 µg/ml for selection. GFP immunofluorescence was assessed by using an Olympus IX71 microscope filtered with 560-nm excitation and 645-nm emission filters. Visible colonies were grown to 80% confluence in the presence of 2 µg/ml puromycin prior to western blot and apoptosis analysis.

### Chromatin immunoprecipitation assay

The chromatin immunoprecipitation (ChIP) experiments were done essentially as previously described with some modifications [55],[56]. Saos-2 cells (10×10^6^) transfected HA-p53 with or without GFP-Gemin3 in the presence of pGL-p53-RE or pGL3-basic vector alone were cross-linked with 1.1% (v/v) formaldehyde, 100 mM NaCl, 0.5 mM EGTA, and 50 mM Tris-HCl (pH 8.0) in growth medium at 37°C for 10 min, then at 4°C for 50 min. Formaldehyde was quenched by adding 0.05 vol 2.5 M glycine. Fixed cells were washed with PBS, incubated for 15 min in 15 ml of 10 mM Tris-HCl (pH 8.0), 10 mM EDTA, 0.5 mM EGTA, and 0.25% (v/v) Triton X-100, followed by 15 min in 15 ml of 10 mM Tris-HCl (pH 8.0), 1 mM EDTA, 0.5 mM EGTA, and 200 mM NaCl, and finally sonicated in 1 ml of 10 mM Tris-HCl (pH 8.0), 1 mM EDTA, 0.5 mM EGTA, 1% (w/v) SDS plus 1 mM PMSF, 1 µg/ml aprotonin, leupettin, and pestatin to an average fragment size of 300–500 bp. 20% of solubilized chromatin extracts were saved for input followed with cross-link reverse step, and the remaining were clarified by centrifugation at 12,000 g, and diluted to 6 OD_260_ U/ml in IP buffer [140 mM NaCl, 1% (w/v) Triton X-100, 0.1% (w/v) sodium deoxycholate, 1 mM PMSF, 100 µg/ml salmon sperm DNA, and 100 µg/ml BSA]; preincubated for 1 h at 4°C with 10 µl/ml 50% (v/v) Protein A-agarose (Invitrogen Life Technologies, Camarillo, CA) with normal mouse/rabbit sera; reconstituted in PBS, and washed several times in IP buffer. Aliquots (600 µl) were incubated with 20 µg of each specific antibody for overnight at 4°C. Immune complexes were separated into bound and unbound complexes with protein A-agarose and cross-links were reversed by treatment at 65°C overnight. After treatment with RNase A and proteinase K, samples were extracted once with phenol/chloroform, and the DNA was precipitated with 2 volumes of ethanol. Precipitated DNA was pelleted, washed once with 70% ethanol, dried, and resuspended in 100 µl of water. The DNA was analyzed by quantitative PCR using Ampicilin primers (forward: 5’-CATCTTACGGATGGCATGAC-3’, reverse: 5’-CAACGATCAAGGCGAGTTAC-3’).

### Colony formation assay

Ten million of Saos-2 cells were typically transfected using electroporation with different combinations of expression plasmids as shown in the text. Transfected cells were cultured in the selection medium (DMEM supplemented with 100 mg/ml G418). After 14 days, cells were fixed on the plates with formaldehyde and stained with 0.1% crystal violet. The amount of the colonies in each dish was scanned by Li-Cor Odyssey and counted. The data are presented as the average from two independent experiments.

### Quantitative real-time PCR

Total RNA from cells was extracted using Trizol reagent and cDNA was made with a Superscript II reverse transcription kit (Invitrogen, Inc., Carlsbad, CA). The primers for real-time PCR were as followings: for p53: 5′-CCT GAGGTTGGCTCTGACTGTA-3′(sense) and 5′-TCCGTCCCAGTAGATTACCAC- 3′ (antisense), yielding a 136-bp product; for p21: 5′-GAGGGCAAGTACGAGTGG CAA-3′ (sense) and 5′- CTGCGCATTGCTCCGCTAACC-3′ (antisense), yielding a 170-bp product; for Bax: 5′- TGCTTCAGGGTTTCATCCAGGA-3′ (sense) and 5′- ACGGCGGCAATCATCCTCTG-3′ (antisense), yielding a 172-bp product; and for GAPDH (glyceraldehyde-3-phosphate dehydrogenase): 5′-CTCCTCTGACTTCAAC AGCG-3′ (sense) and 5′-GCCAAATTCGTTGTCATACCAG-3′ (antisense), yielding a 112-bp product. The cDNA was amplified by using 10 µl of Master Mix from the DyNAmo SYBR green quantitative real-time PCR kit (MJ Research, Inc.), 1 µM of each primer, and 2 µl of the cDNA product in a 20 µl total volume. Thirty cycles of 1 min at 94°C, 30 s at 55°C, and 40 s at 72°C were followed by 10 min at 72°C in an MJ Research Opticon II thermocycler (MJ Research, Inc., Waltham, MA). A melting curve analysis was performed to verify the specificities of the amplified products. The values for the relative levels of change were calculated by the “delta delta threshold cycle” (ΔΔC_T_) method and each sample were tested in triplicates.

### Apoptosis assay

The apoptotic cells of stable Gemin3 and control knock down cells were analyzed by propidium iodide (PI) flow cytometric assay, which is based on the principle that DNA fragmentation and the consequent loss of nuclear DNA content occurs at the late phase of apoptosis. Briefly, 10^6^ cells with serum starvation treatment of 0.1% serum for 12 h were collected and fixed with 100% ethanol for 2 h at 4°C, washed with 1x phosphate-buffered saline (PBS), and stained with 50 µg/ml propidium iodide (Sigma, St. Louis, MO) and 1 µg/ml RNase for 1 hour in the dark at 4°C. The stained cells were subseqeutly analyzed using FACSCalibur cytometer (Becton Dickinson, San Jose, CA) and FlowJo Software (Tree Star, Ashland, OR).
